The article "Recent Progress in Traditional Chinese Medicines and Their Mechanism in the Treatment of Allergic Rhinitis" was retracted in 2023. Reasons: unreliable results or conclusions; concerns about the data; concerns about the peer review; concerns about the citations.

# Recent Progress in Traditional Chinese Medicines and Their Mechanism in the Treatment of Allergic Rhinitis

**DOI:** 10.1155/2022/3594210

**Published:** 2022-04-11

**Authors:** Dehong Mao, Zhongmei He, Linglong Li, Yuting lei, Maodi Xiao, Huimin Zhang, Feng Zhang

**Affiliations:** Department of Otolaryngology, Yongchuan Hospital of Traditional Chinese Medicine, Chongqing Medical University, Chongqing 402160, China

## Abstract

**Objective:**

To conduct a systematic review on the mechanism of action and use of traditional Chinese medicines (TCM) in allergic rhinitis treatment.

**Background:**

Allergic rhinitis (AR) is a type I allergic disease of the immune system induced by immunoglobulin E mediated inflammation and is characterized by sneezing, nasal itching, paroxysmal nasal obstruction, mucosal edema, cough, and rhinorrhea. More than 500 million people have been affected by rhinitis worldwide in the past 20 years, leading to negative effects on health, quality of life, and social relationships. Currently, the trending medicines used in the case of AR include intranasal corticosteroids and oral H1 antihistamines, which are given as combinatorial medicines supplemented with immune therapy. These medications have been found to be very effective in either the short term or long term; however, they have been found to possess some serious side effects. *Search Methodology*. The information in this article on classical and traditional Chinese medications used to treat AR was derived from original papers and reviews published in Chinese and English language journals. Two Chinese databases (Wanfang and CNKI) and three English databases (Cochrane Library, PubMed, and Embase) were utilized for data gathering.

**Results:**

Traditional Chinese remedies have been identified to influence the production of cytokines such as IL-5 and IL-6, which are key mediators of eosinophilic inflammation, TNF-*α*, which stimulates TH2 cells at the site of inflammation, and NF-*к*B, which is required for cytokine and IgE antibody production. TCM has also been shown to be successful in lowering histamine levels, preserving histological changes by decreasing the thickness of the lamina propria, and downregulating the expression of Orai1, STIM1, and TRYC1, showing low expression of Ca^+2^ channel proteins.

**Conclusion:**

In this review, we discussed a series of classical, traditional Chinese medications, including *Centipeda minima*, *Scutellaria baicalensis*, licorice root (*Glycyrrhiza uralensis*), and others, as potential antiallergic agents and investigate their in vivo effect upon the production of cytokines and release of histamines for allergic rhinitis treatment.

## 1. Introduction

Allergic rhinitis (AR) is usually a severe condition that develops due to allergen exposure and results in IgE-mediated inflammation of the nasal membranes. The common symptoms found among patients with AR include sneezing, nasal obstruction, itching sensation in the nasal cavity, and rhinorrhea. These major symptoms may often be accompanied by fatigue from nasal discomfort, itching sensation around the eyes, swelling of the nasal mucosal membranes, postnasal dripping, and cough [1]. On the far current record, approximately 15–20% of the population around the globe is affected by AR, with a dominating ratio in western countries [2, 3]. The treatment of the condition potentially focuses on alleviating the symptoms rather than addressing the root cause of the issue. Hence, patients are often recommended to avoid direct contact with allergens such as pollen, dander, dust mites, and cockroach infestations, which can potentially stimulate the arousal of rhinitis. Considerably, the first line of treatment is solely based on (intranasal antihistamines, corticosteroids, and cromolyn) to reduce inflammation. However, some cases might require surgical intervention [4].

Using the allergen challenge test at the molecular level, several researchers have established that people with AR secrete mediators such as histamine and leukotriene (LT). These proinflammatory factors have been detected in nasal secretions of the affected individuals upon exposure to allergens, but little has been known about their secretion in natural conditions [5–7]. Previous studies have reported the secretion of cytokine (IL-1*α*), a proinflammatory factor, upon exposure to allergens during the early or late phase of the reaction [8–10]. Thereby, it was suggested that the cytokine might have a crucial role in activating endothelial cells long with T-lymphocytes, further stimulating the cytokine release. Recent research has also discovered the presence of IL-1Ra, a naturally occurring inhibitor, in a higher molar concentration in the nasal discharges of AR patients and controls [11]. The antagonist (IL-1Ra) binds with the IL-1 receptor, preventing the active (IL-1*α*) binding without affecting its respective biological response. Similar to IL-1*α*, another chemokine of the interleukin-8 family, interleukin-8 (IL-8), has been found to be elevated throughout the late stages of the disease and is being investigated as a possible candidate in eosinophil movement in certain conditions.

According to a seasonal study conducted to assess the effect of cytokines upon exposure to allergens, it was deduced that a constant incline in the concentration of leukotriene and Eosinophil Cationic Protein (ECP) was prominent throughout the season. According to the findings, histamine concentrations only elevated late in the season and postseasonally. Additionally, the cytokine IL-1*β* and its natural antagonist, IL-1Ra, were assessed. Surprisingly, there was a considerable rise in IL-1*β* concentrations from early in the season to postseason, corroborating the hypothesis of chronic proinflammatory upregulation in seasonal allergic rhinitis. Additionally, the same study determined a considerable decrease in IL-1Ra concentrations during the early season, indicating dysregulation of the local anti-inflammatory capacity. Similarly, nasal secretions contained a significant rise in IL-1*β* concentration, confirming the assumption of chronic proinflammatory regulation.

Along with IL-1*β*, the considerable downregulation of IL-8 and myeloperoxidase indicates disruption of localized immunity, implying a substantial connection between the two variables. Myeloperoxidase is a marker of neutrophil activation, and its lower expression means reduced IL-8 secretion. Since neutrophils account for about 40%–60% of the cells on the mucosal surface and may operate similarly to macrophages, their dysregulation may increase susceptibility to infectious diseases. To summarize, allergic rhinitis does certainly reflect chronic inflammation, as evidenced by eosinophil activity and prolonged elevation of the proinflammatory cytokine IL-1*α*. As a result, the release of cytokines continues for weeks after pollen contact is ceased in persistent and seasonal allergic rhinitis. Numerous components, targets, and mechanisms underlying allergen-induced inflammatory disorders remain unknown despite substantial research on allergic rhinitis. Due to the complexity of the disease, only symptomatic treatment or combined drugs treatment has been recorded to date. Although the following TCM herbs are beneficial against allergic rhinitis, no comprehensive assessment of their anti-allergic-rhinitis mechanisms information from published scientific results has yet been undertaken. As a result, the current study concentrated on using traditional Chinese medicinal herbs to treat AR. This review will cover traditional Chinese medicines (TCM) that are widely used to treat allergic rhinitis.

Studies have demonstrated certain herbs to change biological pathways implicated in allergic rhinitis, such as eosinophil cell death, adhesion molecule modulation, mast cell generation, T_H1_/T_H2_ imbalance, nuclear factor, chemokine concentrations, and IgE regulation [12] (Table 1). Herbs that are frequently used to cure allergic rhinitis comprise *Xanthium* fruit, *Scutellaria* root (*Scutellaria baicalensis*), *Centipeda* herb (*Centipeda minima*), licorice root (*Glycyrrhiza uralensis*), and *Astragalus* roots (*Astragalus membranaceus*). These herbs are the key components in herbal prescription and other Chinese herbs [12].

## 2. *Xanthium* Fructus

The *Xanthii fructus* (XF) is a well-known dried fruit of *Xanthium strumarium*, also called “Cang-Erzi” in Taiwan. It has been used over the years to treat various diseases, including rheumatism, sinusitis, skin pruritus, and headaches (Figures 1(a) and 1(b)) [18]. The *Xanthii fructus* has been shown to reduce mast cell-mediated allergy reactions [19], anti-inflammatory actions in lipopolysaccharide-stimulated inflammatory responses [20], and prevention of *β*-cell damage in type 1 diabetes [21].

As previously stated, allergic rhinitis can be divided into two stages: early and late. The ailment manifests itself within 5–30 minutes of exposure to the antigen, such as mold, dust, or animal dander [22, 23]. Early symptoms following exposure typically include lacrimation, clear rhinorrhea, itching, and sneezing, which are commonly triggered by the production of mast cell secretions, including histamine [24]. On a molecular level, mast cells have been known to play a significant role in inflammatory processes, including the release of proinflammatory cytokines such as tumor necrosis factor (TNF-*α*), interleukin-1*β*, interleukin-8, and interleukin-6 and inflammatory factors including serotonin and histamine (Figure 2) [25–27].

Likewise, the late phase of allergic rhinitis is often characterized by the recruitment of effector cells such as basophils, eosinophils, and T-helper 2 (T_H2_) lymphocytes, causing malaise, irritability, fatigue, and congestion within 6–24 hours after antigen exposure [28–32]. On the other hand, eosinophils have been revealed to play an essential part in the disease's late stage. The abundance of eosinophils in the nasal mucosa of the affected patients indicates the release of proinflammatory mediators such as cysteinyl leukotrienes, eosinophil peroxidase, major basic protein cation in proteins. Presently, the common treatment of AR, as mentioned earlier, includes the usage of corticosteroids, immunosuppressants, and antihistamines. However, their use is restricted due to various adverse effects, such as lipid and glucose metabolism problems, osteoporosis, excessive sedation, and hypertension [33–35].

Over the years, multiple studies have proven the medicinal value of *Xanthii fructus* (XF) with its anti-inflammatory properties. In a survey conducted by An et al., the anti-inflammatory role of XF has been reported on liposaccharide-stimulated mouse peritoneal macrophages [20]. Another study discovered that XF extract shields pancreatic *β*-cells from cytokine-induced damage by inhibiting nuclear factor kappa-B (NK-*к*B) [21]. Another study has established that XF is responsible for inhibiting chronic inflammation found in airways among bronchial asthma patients. Additionally, the extract was found to be effective against histamine and TNF-*α* production in mast cell-mediated allergic responses [19, 36]. We will cover a study paper in this section which examines the mechanism of XF effects by looking at cytokine and caspase-1 levels, the thickness of nasal septum tissue, and the frequency of sneezing behavior in an *in vivo* AR model produced by ovalbumin (OVA). Additionally, the process by which XF inhibits NF-*к*B regulation has been explored.

### 2.1. Effects of *Xanthii fructus* over Nasal Symptoms in Allergic Rhinitis

As discussed earlier, the major symptoms of AR include rhinorrhea, itching, sneezing, and nasal congestion [37]. An OVA-sensitized mouse model was considered to study XF's potential in vivo anti-inflammatory effects. Following sensitization, the extract of XF was injected with cetirizine (a positive control) to assess its anti-inflammatory properties. Compared to OVA-sensitized mice, a model treated with XF had a considerably lower amount of sneezing (*P* < 0.01).

### 2.2. Effects of *Xanthii fructus* on Serum Levels of Histamine, Immunoglobulin E, and OVA-Specific IgE

To investigate the effects of XF, several mice (BALB/c) were injected with OVA injections causing a significant increase in OVA-specific IgE and immunoglobulin E levels. As to our previous understanding, overexpression of IgE is a prominent marker of allergic rhinitis. In OVA-sensitized models, blood levels of histamine and total and OVA-sensitized IgE were observed to be considerably raised with time. However, treatment of mice with XF extract resulted in a significant decrease (*P* < 0.05) in histamine and total and OVA-specific IgE.

### 2.3. Cytokines and the Role of *Xanthii fructus* in Regulation

As we previously understood, cytokines play a vital role in the course of inflammation. The two groups taken under study (i.e., OVA-sensitized mice and mice treated with XF) were observed to understand the trend in the serum level of cytokines. The concentration levels of TNF-*α*, IL-6, IL-5, IF-1*β*, MIP-2, and MIP-1 significantly increased among OVA-sensitized mice. On the contrary, the XF-treated group presented an appreciable decline in the concentrations of these cytokines, indicating its anti-inflammatory function among AR models.

### 2.4. Eosinophil Infiltration and Histological Alterations in the Nasal Mucosa

OVA-sensitized mice groups had extensive eosinophil infiltration in the entire area of the lamina propria, increasing thickness to the nasal tissues, as per histological analyses. However, XF-treated mice groups showed a marked reduction in the thickness of the lamina propria.

### 2.5. Impact of *Xanthii fructus* on the Expression of Caspase-1

Caspase-1 is a member of a protease family also known by the name of IL-1*β*-converting enzyme (IL-1, BCE, or ICE). The enzyme contributes to immune-mediated inflammation by converting the precursor forms of interleukin-1*β* and interleukin-18 into active molecules found in the extracellular compartment [38]. Following the same trend, a significant increase in the expression of caspase-1 was observed among OVA-sensitized mice, whereas, upon treatment with XF, a prominent decrement was noted in the expression of caspase-1.

### 2.6. Mechanism of Action

To our knowledge, allergic illness is mediated by the increase of the Th2 cell subset and the production of particular IgE antibodies by B cells in response to diverse allergens. [39]. In such response, the IgE-sensitized mast cell begins to degranulate, secreting newly synthesized and preformed mediators including cytokines, histamines, cysteinyl leukotrienes, and prostaglandins [40, 41]. TNF-*α* is one of the cytokines that have been shown to have a significant role in allergic inflammation, as it is required for Th2 migration to the site of allergic inflammation and the generation of Th2 cytokines [42]. IL-1*β*, which has mostly been found to be elevated after allergen exposure, activates endothelial cells and T-lymphocytes, leading to further production of cytokines [43].

Similarly, IL-5 and IL-6 have been identified as major mediators of eosinophilic inflammation leading to asthma and are vital in developing nasal secretions, respectively [44]. Asthma patients' bronchoalveolar lavage fluid contains greater levels of the chemokine MCP-1, associated with the activation of eosinophils and basophils [45]. In the absence of an antigen or an anti-IgE antibody, histamine-releasing factors (HRFs) drive mast cells and basophils to release histamine.

Eosinophils move from the blood to the site of inflammation in allergic rhinitis because of the inflammatory stimulus (produced by antigen-presenting cells). This is also one of the main features of allergic rhinitis [46]. Inflammation is frequently reduced when eosinophils are decreased. Now that we know more about caspase-1, an enzyme in the cysteine-protease family, we can better understand how it affects the development of the IL-1 family and how it affects disease-causing immune responses [47]. This thickness of the lamina propria in the nasal septum and infiltration of eosinophils has been found to be conspicuously reduced after treatment with XF.

The expressions of all cytokines predominantly depend on an active transcription factor, NF-*к*B [48]. This activation requires phosphorylation and proteolysis and degradation of I*к*-B*α* (an endogenous inhibitor of NF-*к*B) as its key component [49]. XF was also found to inhibit the phosphorylation and degradation of this transcription factor successfully. Hence, causing the inactivation of NF-*к*B leads to a substantially low level of cytokines. The treatment of AR has led to constructing an animal model in the current research strategy.

In comparison, periodic intranasal OVA treatment has induced typical AR symptoms on a physical and molecular level in the animal models (i.e., inflammatory mediators and IgE production) [48, 50, 51]. XF has drastically decreased levels and an antiallergic impact by blocking the generation of its mediators. Cetirizine, a metabolite that is a selective H1 receptor being used to treat angioedema, urticarial, and allergies [52], has been taken as a positive control. The scheme has also concluded that the effect of XF has been found similar to that of cetirizine.

## 3. Licorice Root

An allergic reaction is mostly regarded as a condition caused by hypersensitivity of the immune system to react with the substances normally considered harmless in all age groups, thereby leading to anaphylaxis [53]. The condition is often mediated by immunoglobulin E response with few medicines available to alleviate the allergic symptoms, including antihistamine drugs (i.e., diphenhydramine, terfenadine, and chlorpheniramine maleate), immune suppressors (hydrocortisone, dexamethasone, and adrenal cortical hormones), and mast cells stabilizers (ketotifen, sodium hydroxypropyl cromate, and disodium cromoglycate). However, as with other drugs, most of these products have been shown to possess side effects. Similarly, symptom relapse has also been observed among patients. In this regard, a suitable alternative derived from food with no side effects may serve as a possible drug of interest to overcome allergic symptoms.

*Glycyrrhiza* is a plant with an ancient origin and has been used over history for herbal medicine and food (Figure 3) [54]. Among other plant constituents, glycyrrhizic acid (GA) is considered one of the main components possessing several pharmacological properties. Numerous research have discovered that biologically active substances in organic foods, such as polyphenols and flavonoids, which have anti-inflammatory or antioxidant properties, lead to antiallergic action. Clinical and experimental studies have revealed the application of glycyrrhizic acid (Figure 4) with its immunomodulatory [55] and anti-inflammatory [56] characteristics. A study reduced asthma-like symptoms in mice with a Balb/c model by taking GA (2.5–20 mg/kg body weight). This was found to be an effective way to treat the mice's asthma, simultaneously preventing the reduction in total IgG2a and interferon-gamma (INF-*γ*) levels. Furthermore, GA (10 mg/kg body weight) has been proven to block the activation of NF-*к*B and STAT-317, hence reducing the onset of acute inflammation. In this section, we will discuss the antiallergic effects of glycyrrhizic acid along with its possible underlying mechanisms.

### 3.1. Through T-Helper Cell Development, GA Plays a Role in OVA-Induced Systemic Allergy Reactions

The antiallergic activity of GA was evaluated in an OVA-induced active systemic allergic response. Conspicuously, multiple allergic symptoms were prominent in the sensitization group, including labored respiration, scratching, and a total decrease in rectal temperature by −1.60 ± 0.1°C. However, the 100 mg/kg body weight group treated with GA showed substantial suppression of allergic symptoms and a net decrease of −0.9 ± 0.1°C in rectal temperature.

The rate of inhibition observed by 100 mg/kg of GA is comparable to that of hydrocortisone, a standard allergy treatment. As for the levels of cytokines, a significant increase was noted among T_H2_ cytokine IL-4, whereas a decreasing trend was prominent among Th1 cytokines (IFN-*γ*) among the OVA-sensitized group. However, after treatment with 100 mg/kg, a significant increase in the level of IFN-*γ* was observed. These findings indicated that an oral dose of 100 mg/kg GA might influence Th1/Th2, resulting in an attenuation of allergic reactions.

### 3.2. Inhibition of OVA-Specific IgE and IgG1 Production via B-Cells

Additionally, the effect of GA on the generation of IgG1 and IgE antibodies in the OVA-sensitized group was studied compared to the controls (*P* < 0.05). The results presented that only 100 mg/kg body weight of GA has significantly decreased the production of OVA-sensitized antibodies (*P* < 0.05). The inhibition effect was found to be similar to that of hydrocortisone. Hence, GA was also found to influence OVA-sensitized antibody-producing B-cells

### 3.3. Role of GA as a “Mast Cell Stabilizer”

According to our prior knowledge, Mast cells contribute to IgE-induced allergy by producing different cytokines, a key cause of allergic conditions. Using passive cutaneous anaphylaxis (PCA) and RBL3-2H3 immunologic cell-based tests, it was further explored if GA can also influence mast cell activation.

The assay results indicate a substantial reduction in the mast cell-dependent PCA reaction in the GA-treated group (in a dose-dependent manner). Similarly, the effect of GA on degranulation was examined by quantifying *β*-hexosaminidase release in the absence and presence of GA. As for the cytokines, glycyrrhizic acid was found to cause substantial suppression in the release of *β*-hexosaminidase from 87.46% to 45.23% with the increment of dosage from 100 to 1000 *µ*g/mL (*P* < 0.05).

### 3.4. Impact of GA upon Expression of Calcium Channel Proteins

According to the available literature, degranulation of RBL-2H3 cells is dependent on the release of Ca^+2^ ions from the endoplasmic reticulum (ER) and the Ca^+2^ ion influx mediated by calcium release-activated calcium channels (CRAC) [57]. Hence, the effect of GA on the influx of Ca^+2^ ions was taken under investigation. The intracellular Ca^+2^ ion concentration was determined using Fluo-3 AM (a fluorescent Ca^+2^ ion indicator). GA at a 1000 *µ*g/mL concentration prevented Ca^+2^ influx mediated by IgE/Ag.

The activation of Ca^+2^ influx-mediated proteins such as stromal interacting molecule 1 (STIM1), Inositol 1,4,5 triphosphate receptor (IP3R), calcium release-activated calcium channel protein 1 (Orai1), and transient receptor potential channel 1 (TRPC1) was also studied. On a similar note, there was a significant decrease in the expressions of Orai1, STIM1, IP3R, and TRPC1 upon treatment with GA. These findings show that GA has no role in the depletion of the ER Ca^+2^ reservoir; instead, the stability of mast cells is predicated on Ca^+2^ influx inhibition due to decreased Orai1, STIM1, and TRPC1) expression.

### 3.5. Mechanism of Action

Glycyrrhizic acid (GA) has been reported to have similar effects on the immune system of Balb/c mice as other natural triterpenoids [58]. These may include anti-inflammatory, antineoplastic, antiviral, immune-regulatory, pharmacological, and antiallergic effects. The three major mechanisms by which antiallergic effect comes into play are (i) a potential role as a mast cell stabilizer, to reduce the secretion of mediators via imparting inhibitory effect over Ca^+2^ influx, (ii) modulation of TH cell development to limit cytokine (IL-4) release from T_H2_ cells, and (iii) influencing OVA-specific antibody-producing B-cells (Figure 5).

According to our previous understanding, GA can decrease serum total IgE and OVA-specific IgE levels [14]. In allergic rhinitis mice models, GA has been shown to elicit a considerable reduction of OVA-specific IgE antibodies in a dose-dependent way. This significant reduction could be caused by blocking T_H1_/T_H2_ differentiation and maturation, which would impede the production of IL-4. Furthermore, GA has also been found to suppress IgG1, later leading to inhibition of basophil activation [59]. Likewise, the study has also presented the role of GA as a mast cell stabilizer, where GA treatment has led to the significant reduction of the intracellular Ca^+2^ levels. As a result, the extracellular process of Ca^+2^ influxes is inhibited. However, no variation in mRNA expression of inositol-3-phosphate receptor was identified in the absence or presence of GA, indicating that GA did not affect endoplasmic reticulum (ER) storage. On the other hand, the expressions of Orai1, STIM1, and TRYC1 were significantly reduced, suggesting that GA may regulate Ca^+2^ degranulation via decreasing calcium channel expression levels.

## 4. *Scutellariae Radix*

*Scutellariae Radix* (RS), also referred to as huangqin in Chinese, is the dry root of the Labiatae plant *Scutellaria baicalensis* Georgi. [60]. In English, the plant is also known as Baikal skullcap or Chinese skullcap, and it is endemic to Asia, particularly Far East Russia, Mongolia, Siberia, East Asia, and China (Figure 6). The plant is frequently used in traditional Chinese medicine to treat cardiovascular and respiratory disorders, gastrointestinal infections, inflammation, and other diseases [61]. Regardless of the whole plant, the usage of RS is more extensive in Japanese and Chinese pharmacopeia with a broad range of therapeutic effects, including detoxifying toxicosis, preventing bleeding and miscarriage, clearing away heat, and moistening aridity [62, 63]. Anti-inflammatory properties of RS have been well documented in *in vivo* and *in vitro* investigations, including inhibition of chemokine, cytokine, and growth factor production from macrophages [64–69], exhibiting potential treatment of colon cancer [70], stroke [71], and colitis [72].

The major biological compounds isolated from RS include phenylethanoid glycosides, flavonoids, diterpenes, triterpenes, phytosterols, polysaccharides, and iridoid glycosides [73]. Among these, over 40 flavonoids along with the form of glycosides have been identified as most abundant [73], which include the key bioactive components oroxylin A-7-glucuronide (OAG), oroxylin A (OA), wogonoside (wogonin-7-glucuronide, WG), baicalein (B), wogonin (W), and baicalin (baicalein-7-glucuronide, BG) [61] (Figure 7).

As previously mentioned, AR is a condition marked by significant pain and other symptoms such as respiratory obstruction, sneezing, congestion, and rhinorrhea, which can lead to ear and nasal abnormalities if left untreated [74]. A complicated allergen-induced inflammatory process within the nasal mucosa causes the condition. On a molecular level, such a process causes the release of histamine and a variety of cytokines and proinflammatory substances, which can trigger vascular dilatation and tear secretion [75]. Among all other activities, the release of IgE has been determined to have a significant part in the overproduction of basophils, eosinophils, and mast cells, as discussed in various sections [76].

Among the various flavonoids mentioned above, baicalein is one of the major constituents of RS found to regulate T_H1_/T_H2_ balance and adjust histamine release from the mast cells [77]. Several research groups have reported the anti-inflammatory role of baicalein in mouse models, alleviating colitis, liver, and vascular inflammation [78, 79] induced by dextran sulfate sodium (DSS) and 2,4,6-trinitrobenzene sulfonic acid (TNBS) [79, 80]. Through an OVA-induced AR animal model, we will explain the regulating efficacy of baicalein derived from RS on clinical symptoms of AR, mucosal histological alterations, and inflammation *in vivo*.

### 4.1. Baicalein's Anti-Inflammatory Properties in AR-Infected Rats

Two major characteristic features, body weight and mass of the vital organs, were considered in OVA group, OVA + baicalein group, and OVA + clarityne group. In terms of body weight, there was no statistically significant difference between the two groups. After 30 minutes of OVA stimulation, the frequency of nasal scratching, degree of nasal outflow, and sneezing pattern in each group were recorded and then overlapped to analyze the findings.

It is worth noting that the OVA-treated group had more sneezing and nasal scratching than the control group. Furthermore, a significant reduction in the frequency of sneeze and nasal grating was found after baicalein treatment, but the inhibition mechanism is still unknown. The primary organ masses (including the spleen, kidney, liver, and heart) were also identified in the OVA-induced, OVA + baicalein-treated, and control groups. The spleen in the OVA-induced group was significantly heavier in comparison to the control group (*P* < 0.05), while the spleen in the baicalein treatment group was considerably lighter in comparison to the OVA-induced group (*P* < 0.05).

### 4.2. The Effect of Baicalein on Inflammatory Variables in AR Rats' Nasal Lavage Fluid and Serum

Levels of inflammatory factors such as IL-6, TNF-*α*, and IL-1*β* were assessed in the OVA-induced (AR model) and baicalein-treated groups better to understand the role of baicalein in inflammatory factor production. In the AR model, there was a considerable increase in IL-6, TNF-*α*, and IL-1*β*, which gradually decreased after treatment with baicalein.

### 4.3. Baicalein's Effect on Inflammatory Cell Infiltration in the Nasal Mucosa and Lung Tissue

Allergen-induced rhinitis, as we all know, results in inflammatory infiltration of the lamina propria. Three groups have been identified based on histological findings using H&E staining. Inflammatory cells were not found in the nasal cavity, lateral nasal walls, or nasal septum in the healthy one. In addition, no signs of vascular congestion or proliferation were observed while presenting normal tissue structure and mucosal glands. However, in the second group (AR model), characteristic changes were present in the histological parameters, including many inflammatory cells (eosinophils, basophils, and mast cells) inside the nasal mucosa. On the other hand, the same feature was significantly reduced in the baicalein-treated group, demonstrating a significant ability to prevent inflammatory cell formation.

Additionally, lung tissue compounds were examined, with pertinent sections stained with H&E to ascertain the extent of lung injury. Damage was visible on the surface, with interstitial edema, thickening, and infiltration of neutrophils into the alveolar wall, as well as the formation of a necrotizing ulcer. However, baicalein was found to alleviate these symptoms significantly.

### 4.4. Baicalein's Effect on p-STAT3 Expression in Nasal Mucosa Tissues

To further validate the impact of baicalein over the inhibition of relevant pathways, the STAT3 signaling pathway was brought into the investigation. According to the findings, baicalein inhibited the phosphorylation of the STAT3 signaling pathway in OVA-induced rats. As discussed earlier, AR can be categorized into two distinct phases. An early stage is usually characterized by IgE-induced activation of inflammatory cells, including neutrophils, eosinophils, and lymphocytes, along with the production of related cytokines (IL1*β*, IL-6, and TNF-*α*). Similarly, the late phase of the condition involves the recruitment of other inflammatory cells such as mast cells and basophils, in addition to the release of chemokines, histamine, and leukotrienes accounting for the anaphylactic shock [81–84]. Typical AR symptoms were reported in this study starting on day 15 and gradually faded after 1.5 hours. According to the present findings, baicalein reduced the frequency of nasal itching and sneezing in AR rats.

## 5. *Centipeda minima*

*Centipeda minima* (L.) A. Braun et Aschers (Compositae), sometimes known as coriander, is an annual herbaceous plant native to eastern tropical zones, Taiwan, and China (Figure 8). The plant, also known as chickweed, is drought-tolerant and spreads throughout China. *C. minima* has been known to possess a spicy taste. It has been traditionally used in Chinese folk medicine to treat sinusitis, relieve pain, reduce swelling rhinitis, and treat cancer for a very long time [86]. Medicinally, the plant has also been used to minimize cough and nasal secretions associated with respiratory complications [16]. To our current understanding, the main medicinal constituents of *C. minima* involved in treatment include polysaccharides, flavonoids, and volatile oils. Pharmacological studies of the plant represent that these therapeutic components have been conventionally used to treat antitumor, antiprotozoal, and allergic rhinitis-associated headaches.

As previously described, allergic rhinitis is a noninfectious inflammation of the nasal mucosa. Symptoms include nasal congestion, runny and itchy nose, and recurrent sneezing episodes. Work and other daily activities may be harmed due to these difficulties. *C. minima* has been demonstrated in studies to decrease eosinophil and mast cell activation, diminish degenerative alterations in nasal mucosal tissues, lower histamine levels, and minimize nasal stiffness [87].

This section will explain the experimental investigation conducted to extract volatile oil components from *C. minima* gathered from seven different geographical sites throughout China and the optimal steam distillation extraction settings. The volatile oil composition of *C. minima* was determined using gas chromatography-mass spectrometry (GC-MS) after extraction. Component-related molecular targets were investigated using network pharmacology analysis. The primary pathways and key targets of *C. minima* components were identified, as well as the overall amount of protein-disease connection. The best volatile oil extraction yield from *C. minima* was obtained at 300°C through a 10-mesh sieve.

### 5.1. Fingerprint and Cluster Analysis

The volatile oil-related GC-MS data from *C. minima* were integrated into the traditional Chinese medicine chromatographic fingerprints similarity evaluation method. The data reveal minor changes in the makeup of *C. minima* samples taken from seven different geographic locations.

The findings reveal that plants collected in Jiangxi, Hubei, Shanxi, and Sichuan have high similarities. We discovered roughly 30 additional volatile oil *C. minima* compounds for each location, 15 of which were identical across all plants.

### 5.2. *C. minima* and Allergic Rhinitis Target Prediction and Mapping

The Venny software tool collected the 15 volatile oil components isolated from *C. minima* specimens in seven geographic areas. 343 relevant targets for 15 components and 2155 diseases targets were identified following a database search. The Venny software was used to import the obtained component targets and disease-related targets. As a result, 117 genes with known intersections were identified. 172 intersection targets were imported into the STRING platform to study protein interactions. The circle's diameter fluctuates according to each protein's degree value, with a higher degree value suggesting that a protein interacts with more pathways. Three proteins were chosen based on their degree and centrality values: mitogen-activated protein kinase 3 (MAPK3), prostaglandin-endoperoxide synthase 2 (PTGS2), and tumor necrosis factor (TNF).

### 5.3. KEGG and GO Analysis

The KEGG and GO analyses of the intersection targets were performed using the R package clusterProfiler. According to the findings of the GO analysis, the biological process (BP) was linked to 1753 pathways, including response to a bacterial molecule, regulation of the inflammatory response, and cellular calcium ion homeostasis, indicating that these genes are involved in related biological processes in vivo and collaborate in the treatment of allergic rhinitis. Our study data revealed 37 cellular components (CC) pathways, including the membrane region, an important part of the resynaptic membrane transcription regulator complex, and other pathways that play a role in allergic rhinitis pathology. KEGG analysis found 137 pathways that were connected. 28 of the target proteins were found to play a role in neuroactive ligand-receptor interaction, 15 of the target proteins are involved in Th17 cell differentiation, and 12 of the target proteins are involved in the VEGF signaling process. The data analysis shows that *C. minima* active ingredients are linked to several possible allergic rhinitis pathways. People who have allergic rhinitis are more likely to get it if they go through the second Th17 cell differentiation process, according to the results of the enrichment analysis and the literature.

### 5.4. H&E Staining

Tissue analysis in rats demonstrated that the nasal mucosa epithelium in the “blank controls” was unaffected. There was no inflammatory cell infiltration in the submucosa of control rats. Cilia were also lost in the disease model group, and the nasal epithelium was damaged. In tissue samples from infected mice, interstitial edema and interstitial inflammatory cell infiltration were observed, as well as gland hyperplasia and swelling. *C. minima* extract-treated rats had much less damage to their nasal mucosa, with less glandular hyperplasia and less inflammatory cell infiltration into the interstitial cell layers in their noses.

### 5.5. ELISA

Immune cells can be activated and regulated by interleukins as second messengers, activating and regulating several inflammatory processes, such as Th17 cell differentiation. Cell proliferation and differentiation can be boosted by TNF, for example. IgE serves as a reference measure for the onset and progression of allergic rhinitis as a key inflammatory factor. Further, we measured the amounts of inflammatory and anti-inflammatory elements (IL-4, TNF-*α*, and IgE) in the serum to verify the network pharmacology's pathway and targets. TNF, IL-2, IgE, and IL-4 were measured in rat serum using ELISA. TNF levels in the model group were substantially higher than those in the control group (*P* < 0.001).

TNF levels were considerably lower in the treatment group compared to the model group (p 0.01). It was found that the IL-2 content in the model group was significantly lower than that in the blank group (*P* < 0.01). There was a statistically significant difference (*P* < 0.01) between the treatment and the model groups in IL-2 levels.

The model group's IL-4 levels were considerably higher (*P* < 0.001). The level of IL-4 in the treatment group was substantially lower than that in the model group (*P* < 0.001). According to the IgE study, the model group had considerably more IgE than the blank group (*P* < 0.001). Compared to the model group, the treatment group had dramatically reduced levels of IgE (*P* < 0.01). Because of this, *C. minima* can reduce inflammatory responses while increasing anti-inflammatory responses. This effect indicates the plant's ability to alleviate the symptoms of allergic rhinitis.

### 5.6. Immunochemistry

Immunohistochemistry results showed that the expression rates of PTGS2 and MAPK3 in inflamed tissues were much greater than those in normal tissues. Compared to the control group, the model group's average optical density of PTGS2 and MAPK3 proteins was significantly higher (*P* < 0.01). There was a big difference in the PTGS2 and MAPK3 proteins in the volatile oil-treated group compared to the model group (*P* < 0.05).

## 6. *Xanthium* Fruit: Emodin

As discussed previously, chronic T_H2_ allergic inflammation such as rhinitis, asthma, and atopic dermatitis affects up to 300 million people worldwide [88, 89]. With the current expansion in urbanization, there is a rise in the number of patients suffering from allergic reactions. There is an urgent need to discover alternative antiallergic medicines that can increase the quality of life while also being safer to use.

Mast cells have long been recognized as a critical player in allergic diseases, where the aggregation of high-affinity IgE receptors (FceRI) on mast cells stimulates the secretion of both preformed (e.g., proteases and histamine) and newly synthesized mediators such as prostaglandin D2 (PGD2) and leukotriene C4 (LTC4) [90, 91]. Signaling cascades are initiated when a cognate antigen (Ag) binds to FceRI. The stimulation of receptor-proximal tyrosine kinases such as Syk, Lyn, Fyn, and Btk and the phosphorylation of other adaptor molecules are examples of these pathways. Syk is essential for the activation of IgE-dependent mast cells. Once active, Syk phosphorylates adaptor proteins such as the linker for activation of T cells (LAT), resulting in the formation of a macromolecular signaling complex that allows for the diversity of downstream signaling required for the creation of various proinflammatory mediators [92–95].

Signaling pathways of such a kind include Ca^+^ ion mobilization mediated through phospholipase C_g_ (PLC_g_), a prerequisite step for LTC_4_ generation and subsequent degranulation [94]. As a result, inhibiting Syk kinase may limit the release of various granule-stored and newly produced mediators [92]. Additionally, crosslinking of FceR1 has been shown to activate the mitogen-activated protein kinase (MAPK), phosphoinositol-3-kinase/Akt (PI3K/Akt), and nuclear factor-*к*B signaling pathways. As a result, several proinflammatory genes, such as those encoding cyclooxygenase (COX-2) and proinflammatory cytokines, are expressed [95].

*Polygonum multiflorum* Thunberg, *Rheum officinale* Bail, *Polygoni cuspidati* (*P. cuspidati*), *radix*, and *Cassia obtusifolia* seed have been utilized in traditional medicines in Eastern Asia for numerous centuries. These oriental plants contain various pharmacological properties, including anti-inflammatory and antiallergic properties [96–99]. Emodin (1,3,8-trihydroxy-6-methylanthraquinone), a compound found in these herbs, has been demonstrated to have a variety of biological actions (i.e., immunosuppressive, antimicrobial, anti-inflammatory, antidiabetic, and antiatherosclerotic activities) (Figure 9) [100–104]. Additionally, Emodin has been shown to inhibit the oncogenic transformation of lung and breast cancer by inhibiting HER2/neu tyrosine kinase activity, indicating its anticancer potential. We will address the antiallergic properties of Emodin and its possible use as a natural remedy for allergic diseases in this part.

### 6.1. Effect of Emodin on Anaphylactic Reaction in Mice

We understand that anaphylaxis is a profound allergic reaction induced by crosslinking specific IgE bound to FceR1. This interaction between FceR1 and IgE stimulates the mediator release from mast cells, causing anaphylaxis [30, 105, 106]. Passive cutaneous anaphylaxis (PCA) and passive systemic anaphylaxis (PSA) were used to assess Emodin's antiallergic activity. PCA was considered in sensitized mice following oral treatment of 25 mg/kg and 50 mg/kg Emodin and 50 mg/kg fexofenadine-HCl for 1 h, via IV challenge with Ag (di-nitrophenyl-human serum albumin in 1% Evans blue dye).

Emodin effectively inhibited the mast cell-dependent PCA reaction in a dose-dependent manner (*n* = 9), suppressing it by 48% (*P* < 0.001) and 55% (*P* < 0.001) at 25 and 50 mg/kg, respectively. PSA levels were determined in mice sensitized with IgE or control saline through IV injection and challenged 24 hours later with an i.v. injection of DNP-HSA. Emodin dose-dependently decreased serum histamine, LTC4, and PGD2 levels (*n* = 9), suppressing LTC4 generation by 38% (*P* < 0.05) and 70% (*P* < 0.05), PGD2 generation by 41% (*P* < 0.01) and 48% (*P* < 0.01), and histamine release by 13.6% (*P* < 0.05) and 34.7% (*P* < 0.01), respectively.

### 6.2. Effect of Emodin on Ca^+2^ Ion Mobilization and Mast Cell Degranulation

The effect of Emodin on the degranulation of mast cells was also examined, considering them to play a major role in anaphylaxis. Initially, the cytotoxic effects of Emodin on bone marrow mast cells (BMMCs) were examined using MTT assay, and no significant effects on cell viability even at 40 mM were observed. As a result, additional studies were conducted at a concentration of <20 mM. To further study the impact of Emodin on IgE/Ag-induced BMMC degranulation, the synthesis of *β*-hexosaminidase (*β*-hex) was evaluated in the presence and absence of Emodin.

A substantial suppression of *β*-hex was observed in a dose-dependent manner (*P* < 0.01). Moreover, the production of cytosolic Ca^+2^ was considered, acknowledging that the release of Ca^+2^ is a key factor in mast cell degranulation [107]. Interestingly, 20 mM of Emodin completely inhibited IgE/Ag-stimulated Ca^+2^ influx (*P* < 0.01).

### 6.3. Effect of Emodin on the Generation of Leukotriene-C_4_ (LTC_4_) from Mast Cells

According to our present understanding, LTC4 production is regulated in two phases (i.e., cPLA_2*α*_ liberation of arachidonic acid (AA) from membrane phospholipids and 5-lipooxygenase oxygenation of free arachidonic acid). In response to increased Ca^+2^ levels, both molecules (cPLA_2*α*_ and 5-LO) translocate from the cytosol to the perinuclear membrane [108, 109].

Furthermore, mitogen-activated kinases (MAPK) phosphorylate cPLA2*α*, a mechanism necessary for optimum arachidonic acid secretion. Further, to assess the mode of action of Emodin, an immunoblot of cPLA2*α*, MAPK, and 5-LO was performed after treatment with IgE/IgA in the presence and absence of Emodin. The obtained results presented that the majority of cPLA2*α* was still in the cytosol regardless of the IgE/Ag stimulation. However, a pool of phosphorylated cPLA2*α* was detected in the nuclear (N-p-cPLA2*α*) and cytosolic (C-p-cPLA2*α*) regions of the activated cells where LTC4 was generated. Under these circumstances, no change was observed in the Lamin B and B-actin (internal control for nuclear and cytosolic fractions, respectively). The IgE/Ag-dependent presence of N-p-cPLA2*α* and C-p-cPLA2*α* was substantially suppressed by Emodin, indicating the potential role of Emodin in the blockage of Ca^+2^-dependent translocation of cPLA2*α* as well as MAPKs (i.e., ERK1/2) dependent phosphorylation.

Similarly, whereas the majority of 5-LO was found in the cytosol (C-5-LO), a small amount was translocated into the nucleus fraction (N-5-LO) upon cell activation, resulting in the formation of LC4. Emodin and each MAPK inhibitor suppressed 5-LO's nuclear translocation effectively.

Immunoblot densitometric measurements have further demonstrated that Emodin reduced the Ag-dependent translocation of cPLA2a and 5-LO from the cytosolic to nuclear fractions. Studies have shown that intracellular Ca^2+^ influx helps regulate 5-LO translocation on multiple occasions [108, 109] and Ca^2+^-independent 5-LO translocation into the nucleus [40]. Though 5-LO can be activated and phosphorylated by MAPKs, [110], it is unclear how MAPK inhibitors prevented 5-LO translocation in IgE/Ag-stimulated BMMCs. There is some preliminary evidence to show that IgE/Ag-activated BMMCs are resistant to intracellular Ca2+ influx when treated with inhibitors of p38 and ERK. Densitometric research indicated that Emodin reduced the activation of all MAPKs evoked by IgE/Ag.

### 6.4. In Mast Cells, Emodin Suppresses Delayed PGD_2_ Synthesis and Cytokine Production

As we are already familiar with the metabolism of arachidonic acid (AA) inside mast cells, the molecule can also opt to alternate COX pathway and thus get metabolism into prostaglandin D_2_ (PGD_2_). PGD_2_ synthesis, in contrast to LTC_4_ synthesis, is a biphasic process. LTC_4_ output and PGD_2_ production occur within a few minutes of each other in the immediate phase of PGD_2_.

The second phase of PGD_2_ synthesis, which lasts for 2–10 hours and is dependent on de novo-induced COX-2, follows the initial phase [17, 85]. IgE-sensitized BMMCs were pretreated with aspirin to eliminate any previous COX-1 activity, followed by a brief wash, and then stimulated with Ag for 7 hours with or without Emodin to examine if COX-2-mediated delayed PGD_2_ production was occurring. Emodin suppressed delayed PGD_2_ production dose-dependently, with a corresponding decrease in COX-2 protein. Since all MAPK inhibitors wiped out COX-2 expression, Emodin's inhibitory impact on MAPKs may be responsible for suppressing COX-2 induction.

Emodin also reduced TNF-*α* and IL-6 production in a dose-dependent manner. It has been found that the NF-*к*B is a key regulator of COX-2 and cytokine expression [111, 112]. The effect of Emodin on the NF-*к*B pathway was studied; results indicated that Emodin significantly inhibited the NF-*к*B pathway by phosphorylating IkappaB kinase (IKK-dependent phosphorylation) and degrading the inhibitory I*к*-B effects on NF-*к*B nuclear translocation.

After IgE/Ag activation, phosphorylation of the IKK complex (p-I*к*Ka/b) and I*к*Ba (p-I*к*Ba) increased, resulting in a decrease in overall I*к*Ba protein and nuclear translocation of NF-*к*B (N-NF-*к*B). Emodin inhibited p-I*к*Ka/b and p-I*к*Ba from increasing, I*к*Ba from decreasing, and N-NF-*к*B from developing. Because Emodin influencess gene transcription in activated mast cells, its effect on the PI3K/Akt pathway was also studied. Emodin inhibited these reactions after IgE/Ag stimulation enhanced the phosphorylation forms of Akt.

### 6.5. Emodin Inhibits Syk Activation

As previously stated, Emodin has demonstrated a highly effective reaction to various mast cell functions. Thus, it would be noteworthy to assess whether it can inhibit an early regulatory step of FceRI signaling. As we know, spleen tyrosine kinase (Syk) plays a key role in initiating FceRI-dependent signaling [92, 93, 95]. Therefore, it would be essential to note whether Emodin affects the inhibition of Syk [96, 113, 114]. In addition, phosphorylated forms of LAT (linker of activated T-cells) and PLC*ɤ*1 (phospholipase C gamma 1) were also considered. These molecules lie downstream of the Syk [115]. The experiment significantly inhibited Syk, LAT, and PLC *ɤ*1 by Emodin. Because PLCg1 phosphorylation is required for inositol phospholipid breakdown and subsequent Ca^2+^ signaling [116], the observed suppression of Ca^2+^ influx by Emodin is most likely due to its inhibitory action on the Syk-dependent activation of PLC1 (Figure 10).

Lastly, to determine if Emodin may also inhibit human mast cell activation, we evaluated its effect on the IgE/Ag-dependent phosphorylation of Syk, PLC*ɤ*1, and LAT in HMC-1 cells. Emodin efficiently suppressed these receptor-proximal events in HMC-1 cells.

## 7. Conclusion

The current review entails a detailed discussion regarding traditional Chinese medicines used to treat allergic rhinitis. The study also outlines the limitation of the currently marketed drugs such as intranasal antihistamines and corticosteroids, which have been shown to possess multiple side effects. On the contrary, Chinese traditional medicines have been found to regulate the production of cytokines, including IL-5 and IL-6, which are the major mediators of eosinophilic inflammation, TNF-*α* which recruits T_H2_ cells at the site of inflammation, and NF-*к*B which is needed for the production of cytokines and IgE antibodies.

Similarly, traditional Chinese medicines (TCM) have also been effective in reducing histamine concentration, maintaining histological changes by reducing the thickness of the lamina propria, and downregulating the expressions of Orai1, STIM1, and TRYC1, indicating the low expression of Ca^+2^ channel proteins. Keeping in view the promising results obtained from TCM, there is a dire need to extend these medications to clinical trials further to reduce the risk ratio of the disease and contribute to society.

## Figures and Tables

**Figure 1:** (a) and (b) Representation of the plant and fruit of *Xanthium strumarium*, also called “Cang-Erzi.”

**Figure 2:** The diagrammatic representation of biomarkers affected during allergic rhinitis.

**Figure 3:** Presentation of a licorice plant [17].

**Figure 4:** Structure of glycyrrhizic acid.

**Figure 5:** The mechanism through which GA exerts its antiallergic impact on IgE-mediated allergic reactions [13].

**Figure 6:** A pictorial presentation of a traditional Chinese medicine herb, Scutellariae Radix [15].

**Figure 7:** Active components obtained from Scutellariae Radix, including flavonoids and glycosides.

**Figure 8:** The plant of *Centipeda minima* [85].

**Figure 9:** Structure of Emodin.

**Figure 10:** Emodin might stop mast cells from getting activated by FceRI. The activation of Syk, a receptor-proximal tyrosine kinase, happens when FceRI comes into contact with the right antigen. A protein called NTAL, which acts as an adaptor, helps Syk control how the PI3K pathway works. This is important because it allows NF-*к*B to make COX-2 and other proinflammatory cytokines. Syk also phosphorylates LAT, which leads to the formation of a macromolecular signaling complex that allows for a wide range of downstream signalings, like PLC1 and Grb2. Activated PLC1 is important for Ca^2+^ responses and activation of PKCs, which are important for degranulation and the movement of cPLA2*α* and 5-LO to the perinuclear membrane and the direction of cPLA2*α* and 5-LO to the perinuclear membrane. The Grb2-mediated pathway is important for cPLA2*α* to be activated properly, leading to eicosanoid hormones [17].

**Table 1:** A cumulative representation of traditional Chinese medicines used to treat allergic rhinitis and the respective pathways and biomarkers regulated by them.

S. no.	Traditional Chinese medicine	Status of biomarkers	Type of study	Techniques/assays used	References
01.	*Xanthi fructus*	TNF-*α*, IL-6, IL-5 ↓	In vivo	Cytotoxicity assay	[13]
		IF-1*β*, MIP-1 ↓		Western blotting	
		MIP-2 ↓		Optical microscopy	
		Histamine, IgE ↓		ELISA	
		Caspase-1 ↓			

02.	Licorice root (glycyrrhizic acid)	IFN-*γ* ↑	In vivo	Evans blue extravasion assay	[14]
		IgE, IgG_1_ ↓		ELISA assay	
		*β*-Hexosaminidase ↓		WST-8 assay	
		IgE mediated Ca^+2^ influx ↓		*β*-Hex assay	
		Orai1, STIM1 ↓		RT-PCR	
		IP3R, TRYC1 ↓		Western blot	

03.	*Scutellaria baicalensis* Georgi.	IL-6, TNF-*α*, IL-1*β* ↓	In vivo	ELISA	[15]
		STAT3 pathway ↓		Immunohistochemical staining	

04.	*Centipeda minima*	TNF-*α*, IL-2, IL-4 ↓	In silico	ELISA	[16]
		PTGS2, MAPK_3_ ↓	In vivo	Immunohistochemical staining, H&E staining	

05.	Emodin	PCA, histamine ↓	In vivo	Evans blue extravasion assay	[17]
		LCT_4_, PGD_2_, LTC_4_ ↓		*β*-Hexosaminidase assay immunoblotting	
		*β*-Hex, Ca^+2^ influx ↓			
		5-LO, MAPK, cPLA2*α* ↓			
		PDG_2_ generation ↓			
		TNF-*α*, IL-6, NF-*к*B ↓			
		Syk, LAT, PLC*ɤ*1 ↓			
		AKT pathway ↓			

## Data Availability

All the data are included in the main text.
